The article "Effect of Muscle Fatigue on Surface Electromyography-Based Hand Grasp Force Estimation" was published in 2021. Journal: Appl Bionics Biomech.

# Effect of Muscle Fatigue on Surface Electromyography-Based Hand Grasp Force Estimation

**DOI:** 10.1155/2021/8817480

**Published:** 2021-02-15

**Authors:** Jinfeng Wang, Muye Pang, Peixuan Yu, Biwei Tang, Kui Xiang, Zhaojie Ju

**Affiliations:** ^1^Department of Information, Wuhan Huaxia University of Technology, 430223 Wuhan, China; ^2^Intelligent System Research Institute, Wuhan University of Technology, 430070 Wuhan, China; ^3^Intelligent System & Biomedical Robotics Group, University of Portsmouth, PO1 3HE Portsmouth, UK

## Abstract

Surface electromyography- (sEMG-) based hand grasp force estimation plays an important role with a promising accuracy in a laboratory environment, yet hardly clinically applicable because of physiological changes and other factors. One of the critical factors is the muscle fatigue concomitant with daily activities which degrades the accuracy and reliability of force estimation from sEMG signals. Conventional qualitative measurements of muscle fatigue contribute to an improved force estimation model with limited progress. This paper proposes an easy-to-implement method to evaluate the muscle fatigue quantitatively and demonstrates that the proposed metrics can have a substantial impact on improving the performance of hand grasp force estimation. Specifically, the reduction in the maximal capacity to generate force is used as the metric of muscle fatigue in combination with a back-propagation neural network (BPNN) is adopted to build a sEMG-hand grasp force estimation model. Experiments are conducted in the three cases: (1) pooling training data from all muscle fatigue states with time-domain feature only, (2) employing frequency domain feature for expression of muscle fatigue information based on case 1, and 3) incorporating the quantitative metric of muscle fatigue value as an additional input for estimation model based on case 1. The results show that the degree of muscle fatigue and task intensity can be easily distinguished, and the additional input of muscle fatigue in BPNN greatly improves the performance of hand grasp force estimation, which is reflected by the 6.3797% increase in R^2^ (coefficient of determination) value.

## 1. Introduction

Surface electromyography (sEMG) is the recording of myoelectric signals of muscle fiber contraction captured by electrodes attached on the surface skin. Due to this electrical manifestation, sEMG has the ability to represent the muscle activation level and contains rich information of muscle force. This ability is widely applied in the accurate estimation of human joint moment which holds significant importance for robot control system design. Human hand grasp force estimation is one of the compelling applications among all of these implementations. The manipulability and dexterity of prosthetic hands, human-assisting devices, and telerobots are facilitated by grasp force estimation. Yamanoi et al. used sEMG signals to determine hand posture and estimate grip force simultaneously for a myoelectric hand [1]. Kim et al. obtained grasp force through upper limb forearm sEMG to control a teleoperation system in real-time [2]. Peternel et al. proposed a muscle fatigue-based method for human-robot collaboration, by which the robot's physical behaviour can be adapted online to human motor fatigue [3]. It should be noticed that the effectiveness and robustness of these applications are depended on the validation of the sEMG-based force estimation which is highly affected by the properties of sEMG signals.

The article "Effect of Muscle Fatigue on Surface Electromyography-Based Hand Grasp Force Estimation" was published in 2021. Journal: Appl Bionics Biomech.

The relationship between sEMG signals and muscle force is mostly extracted by either machine learning-based method or model-based method. Machine learning methods, such as artificial neural network [4] and support vector machines [5], enable the direct mapping from sEMG signals to desired force estimation. The model-based method takes advantage of the musculoskeletal dynamics and incorporates the human knowledge of physiology and motor functionality in an explicit way [6]. The disadvantages of the model-based method are that a general musculoskeletal system modeling for force estimation is still missing which is attributed to the unknown properties, and the corresponding parameters are inherently difficult to identify. Machine learning-based methods mitigate the gap with a compromised yet acceptable interpretability. Among all the modalities, sEMG together with classic regression models has been mostly investigated. Naeem et al. estimated joint force from EMG signals based on a back-propagation neural network (BPNN) [7]. Yang et al. compared different pattern regression methods to optimize the relationship between sEMG signals and hand grasp force [8]. Zhang et al. used linear discriminant analysis (LDA) to realize pattern recognition and artificial neural networks (ANN) to establish the relationship between sEMG signals and fingertip force in each hand grasp modes [9].

Most current research is confined within the improvement of accuracy and reliability for sEMG-based grasp force estimation through a single optimisation of regression algorithms in a laboratory environment instead of a clinical scenario. And the practical factors in clinical settings such as fatigue, sweating, and electrode shift are normally ignored [10]. As one of the most critical factors, muscle fatigue influences the force estimation to a large extent in sEMG-based applications [11]. In daily activities, muscle fatigue leads to failure of force generation to a required value at a normal muscle activation level [12]. When a muscle becomes fatigued, the amplitude-related features of its sEMG signals are notably affected [13]. A typical example is that the root mean square (RMS) of sEMG increases when muscle fatigue happens. In grasp force estimation, RMS is the main feature adopted for EMG-force regression. As a result, the performance of the pretrained force prediction model deteriorates, which is attributed to the unstable RMS representation of sEMG signals. It has been demonstrated that the variant of amplitude-based representation of sEMG-like multiscale RMS (MRMS) gets almost doubled under fatigue condition in a laboratory environment [14]. It is reasonable to incorporate muscle fatigue in sEMG-based grasp force estimation instead of solely depending on the plausible consistency of sEMG signals.

The article "Effect of Muscle Fatigue on Surface Electromyography-Based Hand Grasp Force Estimation" was published in 2021. Journal: Appl Bionics Biomech.

Frequency domain-based method is mostly explored to estimate muscle fatigue from sEMG signals by the analysis of mean frequency (MNF) or median frequency (MDF) [15]. A general conclusion summarises the decreasing shift of MNF or MDF along with the increase of muscle fatigue [15]. Xie et al. applied MNF derived via Hibert-Huang transform to analyse fatigue sEMG signals [16]. Fernando et al. used the ratio of MNF to average rectified value (ARV) as the index of muscle fatigue and muscle fatigue is detected when MNF/ARV falls below a predetermined baseline [13]. Despite the promising results shown by the transition between nonfatigue and fatigue status, the frequency domain metrics exhibit without a determined trend of shifting during singly-fatigue status [17]. An intuitive difficulty brought by this property is seen in the estimation of muscle fatigue using solely frequency metric-based sEMG signal representation. Thus, a more indicative metric is desired to function robustly during the lasting fatigue. The definition of fatigue as any reduction in the maximal capacity to generate force [12] allows the adoption of the loss of maximal voluntary contraction (MVC) to estimate muscle fatigue, where the degree of muscle fatigue is represented by the variant exerted force which is relatively accurate to be measured by additional tangible sensors.

Muscle fatigue has to be taken into account in order to acquire accurate grasp force from sEMG signals. However, so far nobody has been able to explain the relationship between muscle fatigue and sEMG's time-domain features. Even the conclusions of some studies are completely opposite. In this paper, we propose an algorithm to quantitatively estimate the degree of muscle fatigue and evaluate the results by three distinct methods. The substantial effect of muscle fatigue on the performance of hand grasp force estimation is preliminarily demonstrated with experiments on 10 healthy subjects. As the muscle fatigue detection and grasp force estimation are improved, we believe that current applications such as presented in [1–3] will be benefited from our proposed method.

The article "Effect of Muscle Fatigue on Surface Electromyography-Based Hand Grasp Force Estimation" was published in 2021. Journal: Appl Bionics Biomech.

## 2. Forearm Muscle Fatigue Evaluation

Based on the fact that muscle force will decline steadily during a sustained maximal contraction as shown in Figure 1, it is straight to adopt MFL as the index for evaluation of muscle fatigue. In this section, the definition of the proposed force-based metric is given with an emphasis on the case of static contraction for application.

### 2.1. Maximum Force Loss (MFL)

The proposed method to estimate muscle fatigue depends on the measurement of maximal voluntary contraction, which is performed by exerting maximum hand grasp force. To acquire reliable contraction measurement, an easy-to-implement protocol is designed in this paper. At the beginning of a measurement session, the maximum force value is exerted by the subjects and recorded as *MVC_i_*. After repetition of predefined types of static contraction, the force value is recorded for multiple trials as *MVC_t_*. The maximum hand grasp force, as shown in Figure 2, will decrease over contraction tasks and reflects the remained muscle force capacity at the end of each trial. The termination of a session is determined by the failure to accommodate the exertion of required force which indicates that the muscle is too fatigued to accomplish contraction tasks. The required force value is recorded as *MVC_f_*. MFL is finally defined as the following:

(1) $$\begin{array}{c} MFL={MVC}_{i}-{MVC}_{t}, \end{array}$$

where *MVC_i_* and *MVC_t_* correspond to the initial and current MVC force.

To eliminate individual differences, the ratio of the variant maximum hand grasp force to the initial value is adopted as the index of the degree of forearm muscle fatigue, defined as

(2) $$\begin{array}{c} MFL=\frac{{MVC}_{i}-{MVC}_{t}}{{MVC}_{i}}. \end{array}$$

### 2.2. Case Study of Static Contraction

The definition given in the previous section indicates the importance of required force in forearm muscle fatigue estimation. The greater the required force becomes, the less contraction time to maintain the required force level lasts and the muscle is easier to fall into fatigue state. In a case study where subjects perform static contraction tasks by maintaining the required hand grasp force level as steadily as possible, it is necessary to incorporate the influence of required force on muscle fatigue and MFL can be further redefined as

(3) $$\begin{array}{c} MFL=\frac{{MVC}_{i}-{MVC}_{t}}{{MVC}_{i}-{MVC}_{f}}, \end{array}$$

where *MVC_f_* corresponds to the MVC force in the exhausted condition. The proposed muscle fatigue metric MFL can vary from 0 to 1 where 0 indicates the nonfatigue condition and 1 indicates the exhausted condition during static contraction tasks. Equation (3) is adopted together with the assumption of static contraction to estimate muscle fatigue in the following sections.

The article "Effect of Muscle Fatigue on Surface Electromyography-Based Hand Grasp Force Estimation" was published in 2021. Journal: Appl Bionics Biomech.

## 3. Hand Grasp Force Estimation

In this preliminary study, back-propagation neural network (BPNN) is adopted to build sEMG based hand grasp force estimation model.

### 3.1. Experimental Protocol

Ten subjects (seven males and three females, mass 61.1 ± 3 kg, height 1.70 ± 0.03 m, all right-handed) have been recruited in the experiment study. The subjects gave written informed consent before the experiment, and the study was approved by the ethics committee of Wuhan University of Technology. The experiment is conducted with solely nondominant hands, i.e., the left hands, of our recruited subjects, where muscles are more prone to fatigue during the measurement session [18]. The subjects are asked first to seat in a comfortable position with their forearm rest on the table. The sleeve with sEMG electrodes embedded is worn on the subject's forearm with appropriate fixation to avoid the electrode shifting. A hand-muscle developer is held by the subjects' nondominant hand. A pressure sensor is attached to the hand-muscle developer for the measurement of grasp force. With the forearm muscle initially at rest, the captured sEMG with an amplitude at 0 uV is secured prior to the measurement session. Then, the subject is asked to hold the hand-muscle developer in the nondominant hand, with the chair height subsequently adjusted to form an obtuse angle between the forearm equipped with sensor and the upper arm (shown in Figure 3). The sEMG signals are easily interfered by cable movements or the surface electrodes relative movement caused by sleeve slipping ground the forearm. Thus, the subject is required to maintain his posture as much as possible throughout the session to reduce these artefacts.

There are three sessions for one subject to perform: named 50%, 60%, and 70% session. At the beginning of one session, the subject is instructed by visual hints to conduct a 5-second hand grasps at MVC by exerting maximum hand grasp force with the hand-muscle developer, and the force is recorded as *MVC_i_*. Then, a 10-minute rest is provided. After the break, the subject is asked to perform a hand grasp with a muscle contraction at x% *MVC_i_* (*x* = 50, 60, 70, according to which session is performed) as steadily as possible for 10 seconds. This grasp force is recorded as *MVC_f_*. Then, a 5-second grasp at MVC is performed immediately, without a rest, and the maximum hand grasp force is recorded as *MVC_t_*. After that, another loop of 10-second *x*% *MVC_i_* steady contraction and 5-second MVC contraction is performed and repeated multiple times continuously, without a break until *MVC_t_* falls below *MVC_f_*. Then, one session is finished and a 30 minutes rest is given for the purpose of recovering from the muscle fatigue and preparing for the next session. The subject is provided with visual hints throughout the experiments to ensure their adaption to the force variance. The entire experimental procedure of one session is shown in Figure 4.

The article "Effect of Muscle Fatigue on Surface Electromyography-Based Hand Grasp Force Estimation" was published in 2021. Journal: Appl Bionics Biomech.

### 3.2. Data Acquisition

In this study, three muscles closely related to hand grasp are selected to record the sEMG signals, which are palmaris longus, flexor carpiulnaris, and extensor digitorum. A 16-channel electrode-embedded sleeve (ELONXI, UK) is used to cover the aforementioned forearm muscles to collect the sEMG signals where palmaris longus, flexor carpiulnaris, and extensor digitorum mainly correspond to 1-channel electrode, 3-channel electrode, and 5-channel electrode, respectively, as shown in Figure 5. The reference electrode is at the subject's wrist. Before wearing the electrode sleeve, the skin is cleaned by alcohol, and a 10-minute-rest is given after the electrode attachment to improve the contact of the electrode with skin to reduce the resistance within [19]. sEMG signals are amplified by a factor of 5000 with linear range 20 Hz to 500 Hz and sampled at 1000 Hz. The FingerTPS system (Pressure Profile Systems, Inc. (PPS), USA), originally utilised for capturing the tactile force on the finger pulp, is used to measure the hand grasp force in the experiment. Since the finger pulp is not the optimum pressure point during hand grasp, a highly sensitive capacitive-based pressure sensor is fixed to the appointed position on hand-muscle developer (shown in Figure 3). The sample frequency is 100 Hz controlled by the PC clock. The sEMG signals and force measurements are captured and synchronized simultaneously during the experiment.

### 3.3. Data Processing

The relation between sEMG and force signals is extracted in an offline scheme. Two Sallen-Key filters are employed to band-pass filter raw sEMG signals at a bandwidth between 20 Hz and 500 Hz. In addition, a notch filter with central cut-off frequency at 50 Hz (UK power line frequency) is used to remove the power line interference.

The sEMG signals of each channel are segmented by the overlapped windowing technique [20] with a 300 ms window and 100 ms window shift for feature extraction. In this study, RMS and MNF/ARV [21–23] are selected as sEMG features. Except for sEMG signal processing, the mean value of hand grasp force data is adopted in each analysis window.

The article "Effect of Muscle Fatigue on Surface Electromyography-Based Hand Grasp Force Estimation" was published in 2021. Journal: Appl Bionics Biomech.

### 3.4. Force Estimation Methods

BPNN is used to learn the association between sEMG signals and hand grasp forces. In order to evaluate the effect of muscle fatigue on hand grasp force exertion, we propose the following three methods and compare them with locally acquired experiment data.

Time-domain feature driving machine learning-based method (TMLM, as shown in Figure 6): train the BPNN with pooled training data from all muscle fatigue status together. The inputs of BPNN are three muscles' sEMG feature RMS, forming the feature vector

(4) $$\begin{array}{c} \left[RMS_{i\times n}\right], \end{array}$$

where *i* is the channel and *n* is the number of window shift. And the output is the measured hand grasp force. All the data acquired under three distinct hand grasp force levels are formed as the training/testing data for the BPNN.

Combined feature driving machine learning-based method (CMLM, as shown in Figure 7): train the BPNN with combination of time domain and frequency domain features. MNF is often employed for the expression of muscle fatigue information in sEMG-based force estimation. And Japanese researchers further proposed MNF/ARV, which has achieved good results in muscle fatigue detection [13]. So, a combined feature vector is given as

(5) $$\begin{array}{c} \begin{array}{c} \left[{\left({RMS}_{i}\right)}_{n},{\left({MNF}_{i}/{ARV}_{i}\right)}_{n}\right]\\ R^{2}=1-\frac{\sum_{k=1}^{N}{\left(F_{k}-{\overset{\wedge }{F}}_{k}\right)}^{2}}{\sum_{k=1}^{N}{\left(F_{k}-{\bar{F}}_{k}\right)}^{2}}, \end{array} \end{array}$$

where *i* is the channel and *n* is the number of window shift. *F*_*k*_ denotes the actual hand grasp force, ${\hat{F}}_{k}$ is the predicted hand grasp force, ${\bar{F}}_{k}$ is the average of actual hand grasp force, and *N* is the number of testing data.

This method is identical with the above method in output and selection of training/testing data.

Fatigue feature driving machine learning method (FMLM, as shown in Figure 8): train the BPNN with estimated muscle fatigue value as an additional attribute. An additional input of the degree of muscle fatigue estimated by using (3) in combination with the RMS features is provided to the BPNN and expressed as

(6) RMS,i×nMFLi×n,

where *i* is the channel and *n* is the number of window shift. The output and selection method of training/testing data remain the same for all methods, as shown in the following three figures.

The article "Effect of Muscle Fatigue on Surface Electromyography-Based Hand Grasp Force Estimation" was published in 2021. Journal: Appl Bionics Biomech.

All methods adopt the BPNN architecture for force estimation, whose performance is dependent on the choice of network structure, training data, and testing data. The network structure is adjusted by setting different number of nodes from 2 to 20 in the hidden layer with the optimal results [24] provided by a three-layer BPNN. And a Log-Sigmoid function is selected as the transfer function in the network.

(7) $$\begin{array}{c} S\left(x\right)=\frac{1}{1+e^{-x}}, \end{array}$$

where *x* is the input and *e* is the exponential function. Moreover, a four-fold cross validation is adopted to avoid random classification of training data and test data from affecting the prediction results, which helps ensure the reliability and stability of the model.

In this study, *R*^2^ is used to evaluate the estimation performance of three methods, which can be expressed as

(8) $$\begin{array}{c} R^{2}=1-\frac{\sum_{i=1}^{N}{\left(F_{i}-{\overset{\wedge }{F}}_{i}\right)}^{2}}{\sum_{i=1}^{N}{\left(F_{i}-{\bar{F}}_{i}\right)}^{2}}. \end{array}$$

The *R*^2^ can be comprehended as the percentage of the response variable variation that is explained by a linear model [25] and ranges from 0 to 1. In general, the higher the *R*^2^, the better the model fits the data.

*T*-tests were used to verify differences in TMLM, CMLM, and FMLM between different conditions. Differences among subjects are not considered in this paper, as muscle-level dynamic variation is commonly existed. *p* < 0.05 is considered statistically significant for all tests.

## 4. Results and Discussion

In this paper, an algorithm to quantitatively estimate the degree of muscle fatigue is introduced. And the effect of muscle fatigue on hand grasp force estimation is evaluated by conducting three distinct comparison methods. The experimental results of one subject are shown in Figure 9. They are sEMG signals, RMS, and MNF/ARV of three muscles in different levels of static contraction tasks, actual hand grasp force, maximum hand grasp force, and MFL of each sample in different levels of static contraction tasks. These selected features, seen in Figure 10, can basically reflect the force and muscle fatigue information.

### 4.1. Results of Muscle Fatigue Estimation

The experiments last for 300 s, 240 s, and 50 s corresponding to 50% *MVC_i_* (250 N), 60% *MVC_i_* (300 N), and 70% *MVC_i_* (350 N kg) in static contraction tasks, respectively. Figure 10 shows the estimation results of muscle fatigue by the proposed method. Dot arrays of different colors represent the estimation results at different force levels. Through linear fitting, it can be directly seen that MFL grows linearly with the increase of contraction time, which is in accordance with Vøllestad's assumption [12] of muscle fatigue's variety law during a sustained and steady contraction. In addition, the results show that the gradient of time-varying MFL varies at different levels of static contraction. The greater the required force becomes in static contraction, the faster MFL rises, shown in Table 1, which implies that the task intensity can also be distinguished through the proposed metric. The feasibility of the proposed method is recognized in static contraction tasks to estimate muscle fatigue quantitatively.

The article "Effect of Muscle Fatigue on Surface Electromyography-Based Hand Grasp Force Estimation" was published in 2021. Journal: Appl Bionics Biomech.

### 4.2. Results of Hand Grasp Force Estimation

In order to weaken effect of network structure, initial weights, and bias values on the estimation performance, the neural network is retrained ten times at different numbers of nodes (from 2 to 20) in the hidden layer.

In TMLM, we pool training data from all muscle fatigue states to make the network learn the differences among them alone. Predictions of BPNN are shown in Table 2. When the number of node is 4, the mean *R*^2^ is 0.9093, which is the maximum.

In CMLM, we employ MNF/ARV, one feature proposed by Fernando's team for the expression of muscle fatigue information. Predictions of BPNN are shown in Table 3. We set 5 nodes in the hidden layer, and the mean *R*^2^ of prediction results is 0.9255.

In FMLM, we incorporate the quantitative metric of muscle fatigue value as an additional input to explain the effect of muscle fatigue on hand grasp force estimation. Predictions of BPNN are shown in Table 4. The network structure of 10 nodes in the hidden layer brings the maximum mean *R*^2^. Its value is 0.9572.

Comparing the best prediction results of three different methods, as shown in Table 5 and Figure 11, it can be indicated that the mean *R*^2^ obtained in TMLM is 0.9093. It just passes the baseline of applicability (0.9000), which implies the estimation performance of the BPNN model in TMLM is not good enough and predicting model need to be readjusted. In CMLM, the mean *R*^2^ is 0.9255. This shows that employing MNF/ARV proposed by Fernando et al. [13] in sEMG-based force estimation under fatigued conditions is indeed feasible. But it is not an obviously effective approach. Compared with the result in TMLM, *R*^2^ increases by 1.7816%.

As the main work of this study, the estimated muscle fatigue value is used directly as an additional input in FMLM. The results show mean R^2^ can reach to 0.9572, which proves predicting model fits the data very well. It is a great improvement (5.2678%, above 5%, *p* < 0.05) in estimation performance compared with CMLM. It is demonstrated that the additional attribute is an applicable solution to the effect of muscle fatigue on sEMG-based hand grasp force estimation. And MFL proposed in this paper is better than MNF/ARV (*p* < 0.05).

The article "Effect of Muscle Fatigue on Surface Electromyography-Based Hand Grasp Force Estimation" was published in 2021. Journal: Appl Bionics Biomech.

For further explanation, the experimental results of all subjects under different methods are presented as shown in Table 6. Statistics show that the mean *R*^2^ values obtained under the three methods are 0.8656, 0.8919, and 0.9209. Adopting MNF/ARV proposed in [12] for measure muscle fatigue could bring the 3.0383% growth in *R*^2^ in hand grasp force estimation. For comparison, using the MFL proposed in this paper can increase R^2^ by 6.3797%.

The experimental results show that FMLM provides the best estimation performance among the three methods.

## 5. Conclusion

In this paper, we propose an easy-to-implement method to quantitatively estimate muscle fatigue and evaluate the effect of muscle fatigue on hand grasp force estimation. The experiment results demonstrate that the incorporation of muscle fatigue metrics explicitly in the grasp force estimation has a substantial impact on the performance. When estimated muscle fatigue value as an additional input in the machine learning approach, the estimation accuracy improves to a large extent in FMLM. Because the neural network is trained offline and is computationally cheap, the proposed method can be implemented in the current applications, such as in [1–3], as a calibration part to improve the effectiveness and robustness. At the same time, there are still some limitations in this study. During the experiments mentioned above, the degree of the subject's forearm muscle fatigue needs to be estimated at each moment, which requires to intermittently measure the subject's current maximum grasp force. As a result, the force estimation in this work could only be processed offline. So the future work is mainly to address how to estimate muscle fatigue online, that is, how to get MFL online. In fact, the results of this study have provided some potential and guiding ideas for the following work. Under static muscle contraction, the subject's forearm muscle fatigue and muscle contraction time are approximately linear when maintaining a fixed level of hand grasp force. And this linear coefficient seems to have a nonlinear increasing relationship with the target hand grasp force level. Therefore, a nonlinear estimation model of muscle fatigue could be more appropriated in this case, such as

(9) $$\begin{array}{c} MFL=\left(a\times e^{b\times n\%MVC}\right)\times t+c, \end{array}$$

where *n*%*MVC* is the target hand grasp force level. *t* is muscle contraction time. *a*, *b*, and *c* are model parameters.

## Figures and Tables

**Figure 1:** MVC changes during a sustained maximal contraction [12].

The article "Effect of Muscle Fatigue on Surface Electromyography-Based Hand Grasp Force Estimation" was published in 2021. Journal: Appl Bionics Biomech.

**Figure 2:** The measured maximum hand grasp force during a measurement session.

**Figure 3:** Experimental setup.

**Figure 4:** Diagram of the experimental procedure of one session.

**Figure 5:** Diagram of the experimental procedure.

**Figure 6:** Flowchart of grasp force estimation—TMLM.

**Figure 7:** Flowchart of grasp force estimation—CMLM.

**Figure 8:** Flowchart of grasp force estimation—FMLM.

**Figure 9:** Data of static contraction tasks. (a) sEMG signals of three muscles. (b) RMS of three muscles. (c) MNF/ARV of three muscles (d) actual hand grasp force, maximum hand grasp force, and MFL.

**Figure 10:** Muscle fatigue estimation results. Solid lines are linear fitting of the estimation.

**Figure 11:** Single four-fold cross-validation results of each method (a) TMLM. (b) CMLM. (c) FMLM.

**Table 1:** Gradient of MFL.

*MVC_f_*	50% *MVC_i_*	60% *MVC_i_*	70% *MVC_i_*
Gradient	0.0077	0.0108	0.0532

**Table 2:** *R* ^2^ (mean ± sd) of predictions in TMLM.

Number of nodes	2	3	4	5	6
**R** ^2^ **(** **m** **e** **a** **n** ± **sd)**	0.6530 ± 0.0314	0.7037 ± 0.0037	0.9093 ± 0.0205	0.6933 ± 0.0083	0.4682 ± 0.0949
Number of nodes	7	8	9	10	11
**R** ^2^ **(** **m** **e** **a** **n** ± **sd)**	0.8328 ± 0.0095	0.8201 ± 0.0013	0.7978 ± 0.0311	0.7738 ± 0.0183	0.8610 ± 0.0406
Number of nodes	12	13	14	15	16
**R** ^2^ **(** **m** **e** **a** **n** ± **sd)**	0.8259 ± 0.0007	0.7103 ± 0.0074	0.7561 ± 0.0273	0.6653 ± 0.0170	0.6531 ± 0.0713
Number of nodes	17	18	19	20	
**R** ^2^ **(** **m** **e** **a** **n** ± **sd)**	0.7817 ± 0.0211	0.8261 ± 0.0021	0.8156 ± 0.0076	0.8033 ± 0.0145	

**Table 3:** R^2^ (mean ± sd) of predictions in CMLM.

Number of nodes	2	3	4	5	6
*R* ^2^ (mean ± sd)	0.7321 ± 0.0599	0.8357 ± 0.0081	0.7897 ± 0.0276	0.9255 ± 0.0063	0.6594 ± 0.1223
Number of nodes	7	8	9	10	11
*R* ^2^ (mean ± sd)	0.7623 ± 0.0132	0.6229 ± 0.0818	0.6648 ± 0.0049	0.7149 ± 0.0563	0.7281 ± 0.0218
Number of nodes	12	13	14	15	16
*R* ^2^ (mean ± sd)	0.7579 ± 0.0357	0.7932 ± 0.0026	0.5954 ± 0.0214	0.4769 ± 0.1373	0.8362 ± 0.0035
Number of nodes	17	18	19	20	
*R* ^2^ (mean ± sd)	0.7074 ± 0.0104	0.6305 ± 0.0201	0.5928 ± 0.0450	0.7207 ± 0.0422	

**Table 4:** *R* ^2^ (mean ± sd) of predictions in FMLM.

Number of nodes	2	3	4	5	6
*R* ^2^ (mean ± sd)	0.8158 ± 0.0096	0.8663 ± 0.0220	0.8425 ± 0.0055	0.9193 ± 0.0185	0.8356 ± 0.0149
Number of nodes	7	8	9	10	11
*R* ^2^ (mean ± sd)	0.8343 ± 0.0205	0.8795 ± 0.0016	0.8746 ± 0.0127	0.9572 ± 0.0030	0.8842 ± 0.0122
Number of nodes	12	13	14	15	16
*R* ^2^ (mean ± sd)	0.8312 ± 0.0474	0.8652 ± 0.0018	0.8892 ± 0.0017	0.7465 ± 0.1342	0.7358 ± 0.0545
Number of nodes	17	18	19	20	
*R* ^2^ (mean ± sd)	0.8272 ± 0.0143	0.8100 ± 0.0063	0.7836 ± 0.0054	0.8472 ± 0.0010	

The article "Effect of Muscle Fatigue on Surface Electromyography-Based Hand Grasp Force Estimation" was published in 2021. Journal: Appl Bionics Biomech.

**Table 5:** Prediction results of three different methods.

Method	TMLM	CMLM	FMLM
Number of nodes	4	5	10
*R* ^2^ (mean ± sd)	0.8782 ± 0.0005	0.9065 ± 0.0011	0.9506 ± 0.0009

**Table 6:** *R* ^2^ (mean ± sd) of predictions of all subjects under three methods.

Method	TMLM	CMLM	FMLM
Subject 1	0.9093 ± 0.0205	0.9255 ± 0.0063	0.9572 ± 0.0030
Subject 2	0.8910 ± 0.0092	0.9210 ± 0.0039	0.9548 ± 0.0009
Subject 3	0.8255 ± 0.0043	0.8517 ± 0.0064	0.8938 ± 0.0189
Subject 4	0.8224 ± 0.0042	0.8464 ± 0.0049	0.8805 ± 0.0028
Subject 5	0.8286 ± 0.0012	0.8571 ± 0.0014	0.9070 ± 0.0190
Subject 6	0.9293 ± 0.0132	0.9411 ± 0.0209	0.9554 ± 0.0182
Subject 7	0.9199 ± 0.0126	0.9262 ± 0.0050	0.9426 ± 0.0181
Subject 8	0.8802 ± 0.0431	0.9359 ± 0.0088	0.9438 ± 0.0088
Subject 9	0.8153 ± 0.0268	0.8526 ± 0.0131	0.8753 ± 0.0267
Subject 10	0.8350 ± 0.0097	0.8620 ± 0.0130	0.8983 ± 0.0121

## Data Availability

The EMG and force data used to support the findings of this study are available from the corresponding author upon request.
